# Inhibitory receptor immunoglobulin-like transcript 4 was highly expressed in primary ductal and lobular breast cancer and significantly correlated with IL-10

**DOI:** 10.1186/1746-1596-9-85

**Published:** 2014-04-24

**Authors:** Jie Liu, Linlin Wang, Wei Gao, Liwen Li, Xia Cui, Hongyan Yang, Wenli Lin, Qi Dang, Nan Zhang, Yuping Sun

**Affiliations:** 1 Department of Oncology, Jinan Central Hospital, Shandong University, No.105, Jie Fang Road, Jinan, Shandong 250013, PR, China; 2 Department of Pediatric Oncology, Jinan Central Hospital, Shandong University, No.105, Jie Fang Road, Jinan, Shandong 250013, PR, China

**Keywords:** Immunoglobulin-like transcript 4, Interleukin-10, Tumor infiltrating lymphocytes, Immunohistochemistry, Breast cancer

## Abstract

**Background:**

Immunoglobulin-like transcript 4 (ILT4) is an inhibitory molecule involved in immune response and has recently been identified to be strongly inducible by IL-10. The aim of the present study was to examine the associations of ILT4 expression with clinicopathological characteristics and IL-10 expression in primary ductal and lobular breast cancer.

**Methods:**

We studied the expression of ILT4 in 4 cancer cell lines, 117 primary tumor tissues and 97 metastatic lymph nodes from patients with primary ductal and lobular breast cancer by reverse transcription-polymerase chain reaction, western blot or immunohistochemistry analysis. Additionally, IL-10 expression was also investigated using immunohistochemistry in primary tumor tissues. Then the relationship between ILT4 expression and clinicopathological characteristics/IL-10 expression was evaluated.

**Results:**

ILT4 was highly expressed in all 4 human breast cancer cell lines on both mRNA and protein levels. In primary tumor tissues, ILT4 or IL-10 was expressed in the cell membrane, cytoplasm, or both; the positive rate of ILT4 and IL-10 expression was 60.7% (71/117) and 80.34% (94/117), respectively. ILT4 level was significantly correlated with IL-10 (r =0.577; p < 0.01). Furthermore, the expression of ILT4 or IL-10 was associated with less number of Tumor Infiltrating Lymphocytes (TILs) (p = 0.004 and 0.018, respectively) and more lymph node metastasis (p = 0.046 and 0.035, respectively).

**Conclusion:**

Our data demonstrated the association of ILT4 and IL-10 expression in human breast cancer, suggesting their important roles in immune dysfunction and lymph node metastases.

**Virtual Slides:**

The virtual slide(s) for this article can be found here: http://www.diagnosticpathology.diagnomx.eu/vs/1692652692107916

## Background

Breast cancer is one of the most common female malignancies in many countries [1]. Multidisciplinary approaches, including surgery, conventional chemotherapy, radiotherapy, endocrine therapy, bisphosphonates, and HER-2/neu directed therapy, have been used widely for the patients’ treatment; however, a large number of patients responds poorly to these approaches. It is important to expand repertoire of new molecular markers for further therapeutic strategies.

Effective immune response involving T-cell activation defenses normal cells against pathogens through producing cytokines or cytotoxicity. However, immune response to tumor cells is usually inadequate or inactivated, which is one of the most common reasons caused tumor growth, invasion and metastasis [2,3]. Co-stimulatory molecules expressed by antigen presenting cells or tumor cells play a large role in T-cell activation: stimulatory molecules activated T-cell response, and inhibitory molecules suppressed it. When lacking stimulatory molecules (CD80 and CD86) expression or over-expressing inhibitory molecules (B7-H1, B7-H3 and B7-H4) in tumor cells, T-cell is induced to be tolerant or anergic [4,5], which is considered to be associated with immune response escape during cancer development [6-9]. Therefore, studies of co-stimulatory molecules in tumors are not only critical for understanding mechanisms involving in tumor associated immune response, but also helpful for finding new targets of tumor therapy.

Immunoglobulin-like transcripts (ILTs; also referred to as leukocyte immunoglobulin-like receptors) represent a novel immunoglobulin superfamily of both inhibitory and stimulatory receptors involved in immune surveillance [10-12], and are closely related to the killer-cell inhibitory receptor family mapping to the leukocyte receptor complex [13-15]. ILT4, expressed by monocytes, dendritic cells (DCs) and endothelial cells (ECs), has a long cytoplasmic tail containing immunoreceptor tyrosine-based inhibitory motifs which mediates inhibition of cell activation by recruiting tyrosine phosphatase SHP-1 [12,16]. Upregulation of ILT4 on professional and non-professional antigen-presenting cells (APCs) can induce CD4+ T-helper cells anergy; decrease stimulatory molecules expression in T cells [17-19]; and elicit the differentiation of Ag-specific CD4+ and CD8 + Treg cells [20]. In general, the biological function of ILT4 is considered to inhibit the immune response.

The expression of ILTs in cancer cells and their important role in tumor progression become more and more attractive these days. ILT4 is found to be expressed in NSCLC cells [21] with less number of Tumor Infiltrating Lymphocytes (TILs) infiltrated; and the expression of ILT3 or ILT4 in neoplastic B cells is associated with lymphoid tissue involvement in chronic lymphocytic leukemia [22]. However, little is known about the expression and function of ILT4 in other human carcinomas, such as, breast cancers.

IL-10, a pleiotropic cytokine, primarily produced by Th2 cells and Treg cells, has been reported to induce ILT4 upregulation in monocytes and DCs, rendering them tolerogenic [23,24]. Furthermore, in human endothelial cells (ECs), IL-10 also upregulates ILT3/ILT4 expression; and suppresses T-cell co-stimulatory potential of human ECs [25]. However, there is no study to determinate the relationship between ILT4 and IL-10 expression in tumor tissues and assay their role in tumor progression. We here aimed to evaluate the immunohistochemistry expression of ILT4 and IL-10 in a series of invasive ductal and lobular breast carcinomas; analyze the association between ILT4 and IL-10 expression; and discuss their role in breast cancer development through assaying the relationship between ILT4/IL-10 expression and prognostic factors. We hope our findings may be the preliminary experiment for further study on IL-10 and ILT4 function in human breast cancer.

## Materials and methods

### Patient samples

Primary breast cancer specimens were obtained from 117 patients without any preoperative therapy who underwent surgery at Jinan Central Hospital Affiliated to Shandong University, China, between Dec 1st, 2008 and Dec 30th, 2010. All patients signed the informed consent for use of specimens, and the study was approved by the Institutional Review Board (Medical Ethics Committee of Jinan Central Hospital). The median age of patients was 51 years (range, 21 ~ 77 years) at the time of diagnosis. These specimens were 97 invasive ductal carcinomas and 20 lobular carcinomas. Cases with mixed patterns of histologic differentiation were excluded from the analysis. The study also included 97 tumor metastatic lymph nodes from a subset of 12 patients who were from the study group. The tumors were classified as pathologic stage I (33 cases), stage II (52 cases), and stage III (32 cases) using American Joint Committee criterions.

### Cell lines

Human breast cancer cell lines MDA-MB-453, MCF-7, SK-BR-3 and MDA-MB-231 were used in cell experiments. SK-BR-3 and MDA-MB-231 cells were purchased from Cell Resource Center, the Institute of Basic Medical Sciences Chinese Academy of Medical Sciences (Beijing, China). MDA-MB-453 and MCF-7 were conserved in our laboratory. These cell lines were cultured at 37°C in a humidified atmosphere of 5% CO2 in Roswell Park Memorial Institute (RPMI) 1640 medium (Invitrogen, California, USA) supplemented with 10% fetal bovine serum (Invitrogen, California, USA).

### Reverse transcription-polymerase chain reaction (RT-PCR)

Cancer cells were harvested and lysed in total RNA isolation Reagent (RNAiso plus, TaKaRa Biotech, Dalian, China). First-strand cDNAs were prepared with random primers following the instructions of the kit (RNA PCR KIT (AMV) v3.0, TaKaRa Biotech, Dalian, China). RT-PCR involved the primers for human ILT4 5′*GGAGCCTACCCAAAACCC* (forward), 5′ *GTGCGACCACCTGCGATT* (reverse) with use of hot-start Taqgold enzyme (Roche Diagnostic GmbH, Penzberg, Germany). Expression was normalized by β-actin with primers 5′ *GGGACCTGACTGACTACCTC* (forward), 5′ *TCATACTCCTGCTTGCTGAT* (reverse). Cycle conditions were: 94°C, 2 min; 42 cycles for 94°C, 30s; 62°C, 30s; and 72°C, 30s.

### Western blot analysis

Total proteins were extracted from breast cancer cell lines (MDA-MB-453, MDA-MB-231, MCF-7 and SK-BR-3) using RIPA Lysis Buffer (Beyotime, Jiangsu, China) and separated by SDS-PAGE (10%) (Beyotime, Jiangsu, China). These proteins were transferred to 0.45 μm polyvinylidene difluoride membrane (Millipore, Massachusetts, USA) by Bio-Rad transference chamber (Bio-Rad Laboratories, California, USA). Primary antibody to ILT4 (R & D, Minneapolis, USA; dilution 1:500) was used to detect the protein expression. The membrane was incubated with appropriate secondary antibodies labeled to horseradish peroxidase (Santa cruz, California, USA; dilution 1:5000). The protein levels were normalized by reprobing the blots with antibody to β-actin (Santa cruz, California, USA; dilution 1:1000). The signals were detected by the ECL Plus Western Detection Kit (Beyotime, Jiangsu, China) and recorded on the Kodak X-ray films. The protein expression was determined utilizing the BandScan 5.0 software.

### Immunohistochemistry

Immunohistochemical staining was performed as described in our previous studies [9,21]. Briefly, anti-ILT4 mouse monoclonal antibody (R & D, Minneapolis, USA; dilution 1:400), anti-IL-10 mouse monoclonal antibody (Abcam, Massachusetts, USA; dilution 1:100) and anti-CD45RO mouse monoclonal antibody (Abcam, Massachusetts, USA; dilution 1:100) were used as the primary antibodies. Normal mouse IgG was provided as negative control.

### Assessment of Immunohistochemical staining

Immunohistochemical analysis was performed by two independent investigators simultaneously. The percentage of stained cells was recorded at ×400 magnification, in at least 5 random fields. ILT4 and IL-10 expression were evaluated based on the percentage of positive-staining tumor cells [21]. More than 10% of ILT4 brown staining cells was considered as positive while negative (expression <10%). IL-10 expression was divided into high and low group with focal staining intensity more or less than 40%. For studying the relationships between ILT4 and TILs, we counted the number of CD45RO + cells per 1000 total nuclei as described previously [26].

Information on ER, PR, and HER-2/neu status was obtained from the original surgical pathological reports. ER and PR positive staining was defined as staining of >10% of cells. HER-2/neu positivity was defined as 3+ on staining (>30% positive staining of invasive cancer cells) or was determined by fluorescence in situ hybridization (Vysis, Downers Grove, USA) at Quest Diagnostics.

### Statistical analysis

The association of ILT4 or IL-10 expression and clinicopathological variables was analyzed by Chi-square test. The correlation between TILs cell number and ILT4/IL-10 expression was compared by Student’s *t* test. With Spearman correlation coefficient, the relationship of expression between ILT4 and IL-10 was evaluated. p < 0.05 was considered to be statistically significant. Statistical analysis was performed using SPSS v15.0 (SPSS Inc., Chicago, USA).

## Results

### ILT4 expression in human breast cancer cell lines

ILT4 expression in all of the 4 human breast cancer cell lines was found at both mRNA and protein levels by RT-PCR (Figure 1A) and Western blot analysis (Figure 1B), respectively.

**Figure 1:** **ILT4 expression in human breast cancer cell lines. A**: ILT4 mRNA expression was assayed by RT-PCR in breast cancer cell lines. A representative result from 3 independent experiments was shown. **B**: ILT4 protein expression was determined by Western blot analysis. A representative result from 3 independent experiments was shown. β-actin was used as the control.

### ILT4 and IL-10 expression in human breast cancer tissues

The expression of ILT4 and IL-10 in 117 primary tumor specimens was determined by immunohistochemistry. Both ILT4 and IL-10 positive expression were identified in tumor cell cytoplasm, membrane, or both (Figure 2A-B). In normal breast tissues, their expression was absent (Figure 2C-D). Of 117 specimens, the positive rate of ILT4 or IL-10 expression was 60.7% (71/117) and 80.34% (94/117), respectively. Expression of ILT4 was also seen in some stromal macrophages, fibroblasts and plasma cells, and expression of IL-10 was also observed in infiltrating lymphocytes in accordance with previous studies [21,27] (Data was not shown). Furthermore, the expression of ILT4 and IL-10 showed a significant correlation (r = 0.577, p < 0.01; Figure 3A).

**Figure 2:** **Immunohistochemical analysis of ILT4 and IL-10 expression in sections from primary breast cancer (200×). A**: ILT4 positive expression in invasive ductal breast cancer. **B**: IL-10 positive expression in invasive ductal breast cancer. **C**: ILT4 expression was absent in adjacent normal breast tissues. **D**: IL-10 expression in adjacent normal breast tissues was also negative. **E**: ILT4 positive tumor cells in metastatic lymph nodes.

**Figure 3:** **Association between ILT4, IL-10 expression and number of TILs in breast cancer tissues. A**: Correlation between ILT4 and IL-10 expression in breast cancer (r = 0.577, p < 0.01). **B**: The number of CD45RO + TILs was significantly less in ILT4 positive breast cancer tissues than that of negative group (26.71 ± 11.85 and 33.58 ± 13.73, respectively; p = 0.004). **C**: The number of CD45RO + TILs also decreased in IL-10 positive breast cancer tissues compared to negative group (27.65 ± 12.91 and 34.80 ± 14.49, respectively; p = 0.018).

### ILT4 expression in lymph node metastasis

In metastatic lymph nodes, the positive rate of ILT4 expression was 74.2% (72/97) which derived from 12 patients (Figure 2E); and the staining intensity which indicated the expression level was always identical among individual lymph nodes from the same patient. Furthermore, the localization and expression level of ILT4 in tumor cells was similar between primary tumors and corresponding nodal metastasis. Within ILT4-negative tumor metastatic lymph nodes (n = 25), almost all corresponding primary tumors showed negative ILT4 expression except one with 10%-40% ILT4 expression rate in primary tumor.

### Correlation of ILT4/IL-10 expression with the number of TILs

We next assessed the relationship between the expression of ILT4 or IL-10 and the number of TILs in all tumor specimens. Compared to ILT4 or IL-10 negative expression tissues, the amount of TILs seemed to be less in ILT4 or IL-10 positive tissues. The mean number of TILs in ILT4-positive group was 26.71 ± 11.85 and was significantly lower than that in the ILT4-negative group, 33.58 ± 13.73 (p = 0.004; Figure 3B). In addition, the mean TILs number in IL-10-positive group was 27.65 ± 12.91, whereas 34.80 ± 14.49 TILs in IL-10-negative group (p = 0.018; Figure 3C).

### Relationship of ILT4/IL-10 expression with clinical characteristics of breast cancer

As shown in Table 1, expression level of ILT4 or IL-10 was much higher in cases with lymph node metastasis (p = 0.046 and 0.035, respectively). Patients with high expression level of IL-10 were more likely to have advanced disease (stage II-III; p = 0.039) compared to those with IL-10 low expressed. However, no significant correlation was identified between ILT4 expression and tumor stage. Both of ILT4 and IL-10 expressions have no relation with other clinicopathological factors (age, histologic types, grade, tumor size, stages, or receptor status).

**Table 1:** Correlation of ILT4/IL-10 expression with clinicopathologic factors of breast cancer

**Clinicopathologic factors**	**n**	**ILT4 expression**		**p value**	**IL-10 expression**		**p value**
		**Positive**	**Negative**		**High**	**Low**	
**Age**							
≤50	63	40	23	0.502	34	29	0.854
>50	54	31	23		28	26	
**Histologic Types**							
ductal cancer	97	60	37	0.568	53	44	0.432
lobular cancer	20	11	9		9	11	
**Grade**							
I-II	22	10	12	0.105	10	12	0.483
III	95	61	34		52	43	
**Tumor size**							
≤2 cm	50	27	23	0.201	21	29	0.061
>2 cm	67	44	23		41	26	
**Lymph node metastasis**							
N0	43	21	22	**0.046**	17	26	**0.035**
N1-3	74	50	24		45	29	
**TNM stage**							
I	33	16	17	0.09	12	21	**0.039**
II-III	84	55	29		50	34	
**ER**							
positive	82	50	32	0.921	40	42	0.225
negative	35	21	14		22	13	
**PR**							
positive	78	47	31	0.894	38	40	0.239
negative	39	24	15		24	15	
**HER2**							
positive	30	17	13	0.601	11	19	0.055
negative	87	54	33		51	36	

Note: “Bolded values” refer to the statistically significant data.

## Discussion

Cancer is a heterogeneous disease consisting of multiple subgroups with different molecular signatures and clinical behaviors [28,29]. The heterogeneity of breast cancer includes differences in ethnicity, menopausal status, ER/PR status, HER-2/neu expression, and other molecular signatures [30,31]. Finding the sources of breast cancer heterogeneity would contribute to subtype specific therapeutic approaches. ILT4, belonging to the family of immunoglobulin-like inhibitory receptors, plays important roles in modulating the allo-specific antigen immune response to transplants [32]; inducing immune tolerance in pregnancy [33]; and inhibiting myeloid dendritic cell function in HIV-1 infection [34]. And IL-10 is found to regulate the expression of ILT4 in monocytes, DCs and human ECs [24,25]. Besides, emerging evidences suggest that the aberrant expression of ILT4 is involved in tumor progression and lymph node metastasis [21,22]. However, the expression and function of ILT4 in breast cancer and the relationship between ILT4 and IL-10 expression in cancer cells are poorly understood.

In our present study, ILT4 was found to be highly expressed in human breast cancer cell lines, primary tissue specimens and metastatic lymph nodes, while no ILT4 expression was detected in normal breast tissues. It was also expressed in a few macrophages, fibroblasts and plasma cells in breast cancer tissues, which was consistent with the expression pattern in NSCLC tissues [21]. In addition, expression of ILT4 was significantly correlated with lymph node metastasis in clinical breast cancer samples. Previous reports have shown that ILT4 plays an essential role in inducing T-cell anergy, and is necessary for eliciting the differentiation of Ag-specific CD4+ and CD8 + Treg cells [12,17,23]. Furthermore, some studies also revealed that ILT4 was frequently expressed in NSCLC and malignant B cells [21,22], suggesting its important role in tumor cells. Consistent with these findings, our result also showed a large part of breast cancer tissues overexpressing ILT4. ILT4 expressed in tumor cells may act as an inhibitory molecule to suppress the T-cell activity, induce T help cells anergy, or inhibit the differentionation of cytotoxic T cells in microenvironment. It might assist tumor cells in escaping from immune surveillance and facilitate the invasion of tumor cells in lymph nodes. Further studies on detailed mechanisms underlying ILT4 role in human breast cancer warrant further investigation.

Our study further demonstrated that ILT4 overexpression in breast cancer was associated with the overexpression of IL-10. IL-10, a cytokine synthesis inhibitory factor, inhibits T cell or macrophage cytokine synthesis and suppresses their antigen-presenting capacity [35-37]; and was reported to stimulate ILT4 expression through enhancing its promoter activity in human monocytic leukemic cell line THP-1 [24]. IL-10 overexpression in breast cancer confers tumor growth and aggressiveness [38], and is considered as a prognostic indicator for breast cancer [39]. In this study, we found IL-10 expression was not only associated with advanced stage and lymph node metastasis in human primary breast cancer tissues, but also significantly correlated with ILT4 expression (r = 0.577; p < 0.01). Interestingly, the number of CD45RO + TILs in ILT4 or IL-10 positive cancer tissues was less than that of negative groups. CD4 + CD45RO + CD25 + T-cells have been reported to be anergized when IL-10 induces ILT3 and ILT4 upregulation in DCs [23]. We postulated that IL-10 may at least partially regulate the expression of ILT4 in human breast cancer cells; the expression of ILT4 and IL-10 might promote tumor growth and progression by inhibiting the proliferation of CD45RO + TILs and inducing the apoptosis of CD45RO + TILs in the tumor environment. ILT4 and IL-10 may be cooperatively used as predictors of clinical outcomes in breast cancer patients.

In summary, ILT4 was found to be highly expressed in primary human ductal and lobular breast cancer cells, and its expression was significantly correlated with more IL-10 expression, less TILs amount and further lymph node metastasis. Based on previous work and our findings presented here, ILT4 expression in breast cancer may be regulated by IL-10 and promote lymph node metastasis by inducing TILs apoptosis and suppressing T-cell response. However, whether IL-10 upregulated ILT-4 expression through enhancing its promoter activity, and what underlying mechanism of ILT4 and IL-10 act in breast cancer warrant further exploration. Nevertheless, this is the first time to describe the expression of ILT4 and IL-10 in solid tumor cells and analyze the correlation between them. ILT4 may provide a promising target for breast cancer targeted therapy.

## Competing interests

The authors declare that they have no competing interests.

## Authors’ contributions

All authors read and approved the final manuscript. JL and LW designed the study, analyzed the data and drafted the manuscript. WG and LL assisted with the design of the study and collected clinical data. XC, HY, and WL carried out the immunohistochemistry and collected clinical data. QD and NZ performed RT-PCR and Western blot analysis, and involved in pathological diagnosis. YS conceived and designed the study, analyzed the data and edited the manuscript.
